RETRACTED

# Two Myricetin-Derived Flavonols from *Morella rubra* Leaves as Potent *α*-Glucosidase Inhibitors and Structure-Activity Relationship Study by Computational Chemistry

**DOI:** 10.1155/2022/9012943

**Published:** 2022-04-19

**Authors:** Yilong Liu, Ruoqi Wang, Chuanhong Ren, Yifeng Pan, Jiajia Li, Xiaoyong Zhao, Changjie Xu, Kunsong Chen, Xian Li, Zhiwei Gao

**Affiliations:** ^1^Zhejiang Provincial Key Laboratory of Horticultural Plant Integrative Biology, Zhejiang University, Hangzhou 310058, China; ^2^Shandong (Linyi) Institute of Modern Agriculture, Zhejiang University, Linyi 276000, China; ^3^Department of Vascular Surgery, The Second Affiliated Hospital of Zhejiang University School of Medicine, Hangzhou 310009, China

## Abstract

Diabetes mellitus (DM) is a chronic disease characterized by hyperglycemia, and oxidative stress is an important cause and therapeutic target of DM. Phytochemicals such as flavonols are important natural antioxidants that can be used for prevention and treatment of DM. In the present study, six flavonols were precisely prepared and structurally elucidated from *Morella rubra* leaves, which were screened based on antioxidant assays and *α*-glucosidase inhibitory activities of different plant tissues. Myricetin-3-*O*-(2″-*O*-galloyl)-*α*-L-rhamnoside (**2**) and myricetin-3-*O*-(4″-*O*-galloyl)-*α*-L-rhamnoside (**3**) showed excellent *α*-glucosidase inhibitory effects with IC_50_ values of 1.32 and 1.77 *μ*M, respectively, which were hundredfold higher than those of positive control acarbose. Molecular docking simulation illustrated that the presence of galloyl group altered the binding orientation of flavonols, where it occupied the opening of the cavity pocket of *α*-glucosidase along with Pi-anion interaction with Glu304 and Pi-Pi stacked with His279. Pi-conjugations generated between galloyl moiety and key residues at the active site of *α*-glucosidase reinforced the flavonol-enzyme binding, which might explain the greatly increased activity of compounds **2** and **3**. In addition, 26 flavonols were evaluated for systematic analysis of structure-activity relationship (SAR) between flavonols and *α*-glucosidase inhibitory activity. By using their pIC_50_ (-log IC_50_) values, three-dimensional quantitative SAR (3D-QSAR) models were developed via comparative molecular field analysis (CoMFA) and comparative similarity index analysis (CoMSIA), both of which were validated to possess high accuracy and predictive power as indicated by the reasonable cross-validated coefficient (*q*^2^) and non-cross-validated coefficient (*r*^2^) values. Through analyzing 3D contour maps of both CoMFA and CoMSIA models, QSAR results were in agreement with in vitro experimental data. Therefore, such results showed that the galloyl group in compounds **2** and **3** is crucial for interacting with key residues of *α*-glucosidase and the established 3D-QSAR models could provide valuable information for the prediction of flavonols with great antidiabetic potential.

RETRACTED

## 1. Introduction

Diabetes mellitus (DM) is a metabolic disorder characterized by hyperglycemia in the human body. With the changes in lifestyle and improvement of living conditions, the incidence of DM was dramatically raised threatening global human health [1]. Increasing evidence suggests that oxidative stress plays a dominant role in the pathogenesis and development of DM [2]. Many factors such as overnutrition, physical inactivity, impaired glucose tolerance, and inflammatory mediators can induce excessive accumulation of reactive oxygen species (ROSs) or other free radicals during the initiation of DM [3, 4]. Phytochemicals with potent antioxidant activity attract much attention for the prevention and treatment of DM due to its high radical scavenge activity as well as the advantages of safety and good efficacy [5, 6].

*α*-Glucosidase, the carbohydrate hydrolyzing enzyme, hydrolyzes the last step of starch catabolism and releases glucose, which directly affects the blood glucose level in vivo. Inhibition of *α*-glucosidase leads to a delayed glucose absorption in the small intestine and ultimately controls the postprandial hyperglycemia, which is an efficient way for control of DM [7]. Recently, various antioxidants from natural sources were found to possess potent inhibitory effect against *α*-glucosidase [5]. A comparative investigation of 27 dietary flavonoids showed that all these compounds act as *α*-glucosidase inhibitors, among which myricetin was the most potent one [8]. Similarly, myricetin showed the strongest *α*-glucosidase inhibition capacity among 15 flavonoids, followed by fisetin and quercetin [9], which all belong to flavonol subclass of flavonoids. Such results implied that flavonols might be an effective class as *α*-glucosidase inhibitors. However, so far, there has been no systematic study on the structure-activity relationship (SAR) for *α*-glucosidase inhibitory effect of natural flavonols. It was probably due to the huge structural diversity of flavonol compounds and the difficulty in obtaining pure monomers.

As one of the widespread flavonols, myricetin was first isolated from the bark of *Myrica nagi* [10]. Chinese bayberry (*Morella rubra* Sieb. et Zucc.), a kind of berry fruit native to China, also belongs to the Myricaceae family. It is rich in antioxidants including anthocyanins and flavonols [11, 12]. By analyzing the flavonol profiles in different tissues of Chinese bayberry, it is found that tissues with lower anthocyanins, such as bark, leaf, and young fruits, had much higher flavonol contents than mature fruits [13, 14]. Especially in bayberry leaf, the myricetin content is up to 10 mg/g fresh weight (FW) [13].

RETRACTED

Bayberry trees are evergreen throughout the year with luxuriant branches and leaves, which are pruned two or three times a year producing much leaf wastes in the orchard [15]. Accumulating evidence unveiled that flavonol-rich extracts from bayberry leaves exhibited multiple bioactivities such as antioxidative and anti-inflammatory activities [16, 17], suggesting the great utilization potential of bayberry leaves. However, so far, there is no report about the precise preparation and accurate structural elucidation of flavonols in bayberry leaves. Flavonol components in bayberry leaf extracts were tentatively identified [18], which limits the further utilization of bayberry leaves.

In the present study, an efficient protocol was developed for rapid separation of flavonols from bayberry leaves and *α*-glucosidase inhibitory effects of the purified flavonols were tested. For systematic analysis of SAR between flavonols and *α*-glucosidase inhibitory activity, more natural flavonols were analyzed for the function on enzyme activity. Computational chemistry including molecular docking and three-dimensional quantitative SAR (3D-QSAR) was applied to study the binding modes of diverse flavonols to *α*-glucosidase and generate models for search and design of novel *α*-glucosidase inhibitors as therapeutic alternatives for diabetes.

## 2. Materials and Methods

### 2.1. Chemicals

Flavonol standards (HPLC ≥ 95%) were purchased from Shanghai Yuanye Bio-Technology Co., Ltd. (Shanghai, China). Acetonitrile and methanol of chromatographic grade for liquid chromatography-mass spectrometry (LC-MS), as well as *α*-glucosidase from *Saccharomyces cerevisiae* (23 U/mg), acarbose, and p-nitrophenyl-*β*-d-glucopyranoside (PNPG), were obtained from Sigma-Aldrich (St. Louis, MO, USA). Other solvents were all of analytical grade purchased from Sinopharm Chemical Reagent Co., Ltd. (Shanghai, China).

### 2.2. Flavonol-Rich Extracts from Different Bayberry Tissues

Leaves, stem, and young fruits of Chinese bayberry were collected from Lanxi County, Zhejiang Province, China. All materials were transported to the laboratory within 6 hours of sampling and frozen with liquid nitrogen. After being ground into a fine powder, all samples were stored at -80°C before analysis. For the preparation of extracts from different bayberry tissues, each sample powder was extracted twice with an 80% aqueous methanol as material-to-solvent ratio of 1 : 10. It was stirred well and sonicated for half an hour with ultrasonic power of 30 W and ultrasonic frequency of 60 kHz. After centrifugation at 10,000 rpm for 10 min, the supernatants were obtained as the extracts from bayberry leaf, stem, or young fruit pulp for further experiments.

RETRACTED

### 2.3. Determination of Antioxidant Activity

Chemical antioxidant capacities including 1,1-diphenyl-2-picrylhydrazyl (DPPH) free radical scavenging activity, 2,2′-azinobis(3-ethylbenzothiazoline-6-sulfonic acid) (ABTS) radical scavenging activity, and ferric ion reducing antioxidant power (FRAP) were measured according to previous report [19]. Ascorbic acid (Vc) was used as the control. Results were calculated by the standard curve method and expressed as milligrams of Vc equivalents per gram FW (mg VcE/g FW). Each experiment was repeated three times.

### 2.4. Determination of *α*-Glucosidase Inhibition

Inhibitory effects of flavonol-rich bayberry extracts or flavonols on *α*-glucosidase were detected as our previous report [20]. In the reaction, 20 *μ*L *α*-glucosidase of 0.2 U/mL in 0.1 M potassium phosphate buffer (PPB, pH 6.8), 112 *μ*L of 0.1 M PPB, and 8 *μ*L of test sample were preincubated in the 96-well microtiter plate at 37°C for 15 min. Then, 20 *μ*L PNPG of 2.5 mM was added to each well and incubated for another 15 min at 37°C. Finally, the reaction was terminated with the addition of 80 *μ*L Na_2_CO_3_ of 0.1 M, and absorption value (OD) was measured at 405 nm by a microplate reader (Thermo Electron Co., Vantaa, Finland). Acarbose and DMSO were used as the positive and negative control, respectively. Reaction solution without enzyme was used as a blank. The calculation formula was as follows:

(1) $$\begin{array}{c} \alpha -\text{Glucosidase inhibition rate }\left(\%\right)=\left(1-\frac{{\text{OD}}_{\text{sample}}-{\text{OD}}_{\text{sample blank}}}{{\text{OD}}_{\text{control}}-\text{O}{\text{D}}_{\text{control blank}}}\right)\times 100. \end{array}$$

The value of half maximal inhibitory concentration (IC_50_) represented the extract (*μ*g/mL) or flavonol (*μ*M) concentration when its inhibition rate reaches 50%. Such value was calculated based on the dose-dependent inhibitory rate of the test sample against *α*-glucosidase.

### 2.5. Isolation and Purification of Flavonols from Bayberry Leaves

Efficient simultaneous purification procedure of flavonols from bayberry leaves was established by solid-phase extraction combined with high-speed counter-current chromatography (HSCCC) and semipreparative HPLC (pre-HPLC). Bayberry leaves were frozen in liquid nitrogen, freeze-dried (FM 25EL-85, VirTis, Gardiner, NY, USA), and then ground into a fine powder. The lyophilized powder of bayberry leaves was extracted three times by 80% aqueous methanol with a solid-to-liquid ratio of 1 : 10. The mixture was sonicated for 30 min and filtered by a Buchner funnel with Whatman No. 1 filter paper. The combined filtrate was evaporated at 37°C under reduced pressure by a rotary evaporator (Concentrator Plus, Eppendorf, Germany) to remove methanol. The remaining aqueous extract solution was centrifuged at 10,000 rpm for 10 min at room temperature. The supernatants were loaded to the Sep-Pak® C18 cartridge (12 cc/2 g, Waters, Milford, MA, USA) that was activated with 4 bed volumes (BV) of methanol and conditioned with 4 BV of ddH_2_O. Then, the cartridge was washed with another 4 BV of ddH_2_O and 4 BV of 2% aqueous methanol to remove impurities and eluted with 12 BV of 30% methanol and 6 BV of 40% methanol. Each eluent was vacuum-dried to obtain 30% fraction and 40% fraction for further purification.

RETRACTED

Compound **1** was purified from the 30% fraction by HSCCC (TBE 300A, Tauto Biotech., Shanghai, China) combined with a TBP5002 pump and a TBD2000 UV detector. Petroleum ether-ethyl acetate-methanol-water (2 : 6 : 2 : 5, *v*/*v*/*v*/*v*) were selected as the solvent system, where the partition coefficient (*K*) of compound **1** was 1.00. Two liters of solvents was put into a separating funnel according to the selected ratio. After equilibrium for an hour, the two phases were separated and degassed by sonication for 30 min. Firstly, the upper phase was injected with the flow rate of 30 mL/min to fill the three polytetrafluoroethylene coil separation columns of HSCCC. The total volume of the columns is 315 mL, and the tube diameter is 1.6 mm. Then, the revolution speed was set as 900 rpm and the flow rate was changed to 3 mL/min. After reaching the set speed, the lower phase was pumped into the separation column until equilibration. The 30% fraction powder was dissolved in the lower phase with the concentration of 20 mg/mL, and the solution was injected through a 20 mL sample loop. Effluent was monitored by the UV detector at 350 nm and collected in every 2 min for a tube for HPLC detection. Finally, tubes with pure compound **1** were combined and vacuum-dried.

Compounds **2** to **6** were purified from the 40% fraction by pre-HPLC consisting of a 2707 autosampler, a 2535 pump, a 2998 detector, and a Waters SunFire prep C18 OBD column (5 *μ*m, 19 mm × 250 mm). The mobile phase solution consisted of ddH_2_O with 0.1% (*v*/*v*) formic acid (A) and 0.1% formic acid: acetonitrile (1 : 1, *v*/*v*) (B). Elution gradient was as follows: 0-10 min, 20%-80% of B; 10-30 min, 80%-100% of B; and 30-35 min, 100%-20% of B. Sample concentration was 150 mg/mL, injection volume was 300 *μ*L, and flow rate was 5 mL/min. Effluent with pure target compound was collected according to the chromatogram at 350 nm.

RETRACTED

### 2.6. Structural Characterization

Structural characterization of flavonols in bayberry leaves was conducted by HPLC, LC-MS, and Nuclear Magnetic Resonance (NMR) Spectroscopy. The operated HPLC system was equipped with a e2695 pump, a 2998 diode array detector, and a SunFire C18 analytical column (5 *μ*m, 4.5 × 250 mm) (Waters, USA). The mobile phase solution was the same as that of pre-HPLC. Gradient program was as follows: 0-40 min, 10%-38% of B; 40-60 min, 38%-48% of B; 60-70 min, 48%-100% of B; 70-75 min, 100%-10% of B; and 75-80 min, 10% of B. Flow rate was set at 1 mL/min, and injection value was 10 *μ*L.

LC-MS identification was carried out as our previous report [11]. Chromatographic separations were performed under the same gradient procedure as HPLC using an Agilent 1290 Infinity system (Agilent Technologies, USA) equipped with an X-Bridge C18 analytical column (4.6 × 250 mm). MS analysis was conducted by an Agilent 6460 triple quadrupole mass spectrometer coupled to an electrospray ionization source (Agilent Technologies, Santa Clara, CA, USA) and operated in the negative ionization mode.

The ^13^C-NMR spectra were measured in DMSO-*d6* at 25°C on an Agilent 600 MHz instrument. Solvent residual peak *δ* 39.52 was used to calibrate all ^13^C chemical shifts in the present study. The chemical shifts of NMR were calculated and extracted by MestReNova (version 6.1.0).

### 2.7. Homology Modeling and Molecular Docking

The 3D structure of *α*-glucosidase from *Saccharomyces cerevisiae* was established by homology modeling using SWISS-MODEL (https://swissmodel.expasy.org/) according to the workflow described by previous report [21]. The amino acid sequence of MAL32 was obtained from the database of NCBI (https://www.ncbi.nlm.nih.gov/protein/) and uploaded in the SWISS-MODEL server to search template. The protein 3AJ7 was found to share high sequence similarity of 72.51% with *α*-glucosidase and used as the template for homology modeling. The structures of diverse flavonols were downloaded from the PubChem database (https://pubchem.ncbi.nlm.nih.gov/). Energy minimization was conducted for each small molecule by MM2 force field in Chem3D 20.0 with the root mean square gradient set as 0.001. Structures were removed water molecules, added hydrogen atoms and Gasteiger charges, and were written as pdbqt files by AutoDockTools [22]. AutoDock Vina was used for the docking simulation of flavonols and *α*-glucosidase [23]. Grid box for *α*-glucosidase was set as 60 × 60 × 60 Å, centered at *X* = 2.900, *Y* = −4.660, and *Z* = 20.039. Intermolecular interaction analysis and molecular visualization were carried out using Discovery Studio 2017 R2 and PyMOL (The PyMOL Molecular Graphics System, Version 2.0.6 Schrödinger, LLC).

RETRACTED

### 2.8. Data Sets

IC_50_ values of the inhibition effects of the tested 26 flavonols on *α*-glucosidase were converted to pIC_50_ values (−log [IC_50_ (*μ*M)∗10^−6^]), which were dependent variables in 3D-QSAR analyses. The training set, comprising twenty-one compounds selected randomly, was used to construct 3D-QSAR models, and the test set, consisting of the remaining five compounds, was applied to evaluate the predictive capacity of the resulting models.

### 2.9. Molecular Alignment

All small molecules were energetically minimized by the method of Powell, force field of Tripos, and charge of Gasteiger-Hückel in SYBYL-X 2.0 (Tripos, Inc., St. Louis, MO, USA) [24]. Max iterations were 10,000, and termination was set as the convergence criterion of 0.005 kcal/(mol∗Å). Other parameters were the default values. Then, molecular alignment was performed using the mother ring of flavonols as the common skeleton, which is a vital step in generating 3D-QSAR models. Compound **2** was selected as the template molecule for its strongest *α*-glucosidase inhibitory effects among all of the tested compounds.

### 2.10. 3D-QSAR

In the present study, 3D-QSAR models of flavonols as *α*-glucosidase inhibitors were established by two methods including comparative molecular field analysis (CoMFA) and comparative similarity index analysis (CoMSIA). In CoMFA, it contained descriptors of steric and electrostatic fields, and field energies were calculated via the probe of a sp^3^ carbon possessing a charge of +1. In CoMSIA, it had three more descriptors including hydrophobic, hydrogen bond donor, and hydrogen bond acceptor fields compared to that of CoMFA, and calculation was performed based on the function of Gaussian-type distance.

Partial least squares (PLS) analysis was applied to establish statistically significant 3D-QSAR models using two and five variables stemmed from CoMFA and CoMSIA descriptors, respectively [25]. Cross-validation was conducted through the leave-one-out (LOO) option, wherein the optimum number of components (ONC) and value of cross-validated coefficient (*q*^2^) were acquired. Finally, the 3D-QSAR models were established after performing the non-cross-validation, by which the coefficient (*R*^2^), *F* test value (*F*), and standard error of estimation (SEE) were obtained.

### 2.11. Model Validation

A high value of *q*^2^ (0.5 < *q*^2^ < 1) is important for the good predictability of the model. In addition, validation of the generated 3D-QSAR models was performed by internal and external validation methods. Internal validation was conducted by predicting the pIC_50_ values for the training set in CoMFA or CoMSIA analysis. The predicted pIC_50_ for the test set were also calculated as external validation, and the predictive correlation coefficient (*r*^2^_pred_) was used to assess the robustness and accuracy of each model.

RETRACTED

### 2.12. Data Analysis

Data expressed as means ± standard deviation (SD) were obtained from three replications. 3D-QSAR statistical results were acquired from SYBYL-X 2.0. IC_50_ values were calculated by SPSS 19.0 (IBM, Armonk, NY, USA).

## 3. Results

### 3.1. Bayberry Leaf Is Screened for Significant Antioxidant Activity and *α*-Glucosidase Inhibitory Effect

Chemical antioxidant assessments combined with in vitro test on *α*-glucosidase are the common methods for the preliminary evaluation of antidiabetic potential, which have the advantages of rapidity and simplicity. Antioxidant capacity of methanol extracts from bayberry leaf, stem, and young fruits was evaluated by chemical methods including DPPH, FRAP, and ABTS assays. Results showed that leaf extract had the significantly higher antioxidant activity than that of stem or young fruit extract as exhibited in all of the three methods (Figure 1(a)). Bayberry leaf extracts also showed stronger inhibitory effect against *α*-glucosidase with an IC_50_ value of 127.37 *μ*g/mL, compared to that of stem (169.29 *μ*g/mL) or young fruits (1134.58 *μ*g/mL) (Figure 1(b)). Such results indicated the greater potential of bayberry leaf for developing *α*-glucosidase inhibitors.

### 3.2. Six Flavonols Are Purified and Precisely Characterized in Bayberry Leaf

As shown in Figure 1(c), six pure flavonols were isolated from bayberry leaf through ultrasonic-assisted extraction and solid-phase extraction combined with HSCCC and Pre-HPLC. By matching the retention time, spectrum information, and MS^n^ spectral data with authentic standards, compounds **1**, **4**, **5**, and **6** were identified as myricetin-3-*O*-rhamnoside (myricitrin), quercetin-3-*O*-galactoside (hyperoside), quercetin-3-*O*-glucoside (isoquercitrin), and quercetin-3-*O*-rhamnoside (quercitrin), with the contents of 9.42 ± 0.36, 0.29 ± 0.01, 0.02 ± 0.00, and 0.24 ± 0.01 mg/g FW, respectively.

Compounds **2** and **3** were isomers as shown in the same precursor ion [M-H]^−^ at *m*/*z* 615.10 (Figure 2). It generated a product ion at *m*/*z* 463 [M-H-152]^−^ by the release of a galloyl moiety. Base peak at *m*/*z* 317 [M-H-152-146]^−^ confirmed the myricetin aglycone and corresponds to the cleavage of the galloyl and a deoxyhexose moiety. Due to the absence of commercial standards, these two compounds were relatively quantified based on the level of compound **6**, contents of which were calculated as 0.20 ± 0.03 and 0.05 ± 0.01 mg/g FW. Further structural confirmation of compounds **2** and **3** was conducted by high-resolution mass (Supplementary Figures 1 and 2) and NMR (Supplementary Figures 3 and 4).

RETRACTED

*Myricetin-3-O-(2* ^″^ *-O-galloyl)-α-l-rhamnoside (**2**)*. ^13^C NMR (151 MHz, DMSO-*d6*) *δ* 177.44 (C-4), 164.94 (COO), 164.19 (C-7), 161.25 (C-5), 157.49 (C-2), 156.39 (C-9), 145.78 (C-3′/5′), 145.44 (C-3^‴^/5^‴^), 138.53 (C-4^‴^), 136.55 (C-4′), 133.32 (C-3), 119.38 (C-1′), 119.24 (C-1^‴^), 108.84 (C-2′/6′), 107.93 (C-2^‴^/6^‴^), 103.97 (C-10), 98.70 (C-6), 98.33 (C-1^″^), 93.54 (C-8), 71.75 (C-4^″^), 71.68 (C-2^″^), 70.65 (C-5^″^), 68.55 (C-3^″^), and 17.56 (C-6^″^).

*Myricetin-3-O-(4* ^″^ *-O-galloyl)-α-l-rhamnoside (**3**)*. ^13^C NMR (151 MHz, DMSO-*d6*) *δ* 177.78 (C-4), 165.70 (COO), 164.30 (C-7), 161.30 (C-5), 157.63 (C-2), 156.47 (C-9), 145.81 (C-3′/5′), 145.38 (C-3^‴^/5^‴^), 138.27 (C-4^‴^), 136.50 (C-4′), 134.85 (C-3), 120.00 (C-1^‴^), 119.61 (C-1′), 108.99 (C-2′/6′), 107.93 (C-2^‴^/6^‴^), 104.03 (C-10), 102.71 (C-1^″^), 98.70 (C-6), 93.57 (C-8), 73.90 (C-4^″^), 70.87 (C-2^″^), 68.61 (C-3^″^), 67.78 (C-5^″^), and 17.46 (C-6^″^).

### 3.3. Different Fractions and Six Purified Flavonols from Bayberry Leaf Show Good Dose-Dependent Inhibition on *α*-Glucosidase

Through the solid-phase extraction, 30% fraction rich in compound **1** and 40% fraction containing compounds **2** to **6** were obtained from bayberry leaf extracts. Results showed that both 30% and 40% fractions had significant inhibition activity on *α*-glucosidase in a dose-dependent manner, with the IC_50_ values of 0.49 *μ*g/mL and 0.71 *μ*g/mL, respectively, which were markedly lower than those of acarbose (IC_50_ = 238.33 *μ*g/mL) (Figure 3). It indicated that the components in each fraction might be potent *α*-glucosidase inhibitors.

Among the six purified flavonols, compound **2** showed the highest *α*-glucosidase inhibition capacity with the IC_50_ value of 1.32 *μ*M, followed by compound **3** of 1.77 *μ*M, which was about 200 times lower than that of acarbose (IC_50_ = 369.15 *μ*M) (Figure 3). For another four compounds, they also had good dose-dependent inhibitory effects against *α*-glucosidase, although the IC_50_ values were relatively higher, and in the order of compounds **1** (IC_50_ = 776.93 *μ*M), **6** (IC_50_ = 1038.97 *μ*M), **4** (IC_50_ = 1148.19 *μ*M), and **5** (IC_50_ = 1195.95 *μ*M) (Figure 3).

RETRACTED

### 3.4. More Natural Flavonols Are Introduced for SAR Study on Flavonols and *α*-Glucosidase Inhibition

In order to explore the SAR between different flavonols and *α*-glucosidase inhibitory activity, besides the six purified flavonols from bayberry leaf, there are more natural flavonols tested including six flavonol aglycones, one myricetin glycoside, six quercetin glycosides, five kaempferol glycosides, and two isorhamnetin glycosides. Chemical structure information of all the tested flavonols and their IC_50_ values for *α*-glucosidase are listed in Table 1.

Six flavonol aglycones showed remarkable *α*-glucosidase inhibitory effects in the order as follows: myricetin (21, IC_50_ = 15.61 *μ*M) > quercetin (22, IC_50_ = 35.39 *μ*M) > kaempferol (23, IC_50_ = 71.00 *μ*M) > fisetin (24, IC_50_ = 86.34 *μ*M) > herbacetin (25, IC_50_ = 123.12 *μ*M) > isorhamnetin (26, IC_50_ = 319.54 *μ*M), all of which are more potent *α*-glucosidase inhibitors in comparison with acarbose (IC_50_ = 369.15 *μ*M) (Table 1). Among the remaining twenty flavonol derivates, IC_50_ values of glycosylated flavonols ranged from 419.60 *μ*M to >2000 *μ*M, which are all higher than those of the corresponding aglycones and acarbose (Table 1). Notably, the gallated flavonol glycosides, i.e., compounds **2** and **3**, possessed the top two lowest IC_50_ values among all of the tested flavonols, as 1.32 and 1.77 *μ*M, respectively, indicating the stronger *α*-glucosidase inhibitory effects than that of flavonol aglycones and glycosides as well as acarbose. The above results demonstrated that the glycosylation modification of flavonols decreased the inhibition capacity, while galloylation of flavonols significantly improved the inhibitory activity against *α*-glucosidase.

### 3.5. Binding Patterns of Diverse Flavonols to *α*-Glucosidase Are Visually Analyzed by Molecular Docking Simulation

Docking analyses were performed to investigate the binding modes and forces between diverse flavonols and *α*-glucosidase. Among all of tested flavonols, the most potent *α*-glucosidase inhibitor, i.e., compound **2**, fitted well to the binding pocket of enzyme (Figure 4), with a predicted binding energy of -10.9 kcal/mol. Its chemical structure consists of the aglycone myricetin, a rhamnosyl and a galloyl moiety.

As shown in Figure 5, aglycone of compound **2** formed Pi-Pi stacked with residue Phe157 and hydrophobic (Pi-alkyl) interaction with Ala278 and Leu218 at its A and C rings. Electrostatic (Pi-anion) interaction was generated with Asp349 at the B ring. Pi-alkyl was also formed between the methyl group of rhamnose ring and Arg312. Notably, the galloyl moiety of compound **2** occupied the opening of the cavity pocket of *α*-glucosidase (Figure 4), along with the Pi-anion interaction with Glu304, Pi-Pi stacked with His279 (Figure 5), and hydrogen bond generated between the O atom of its carbonyl group and Asn241. Such binding orientations might greatly contribute to the strong inhibitory effect of gallated flavonols, as shown in basically the same binding pattern of the galloyl moiety of compound **3**, the second strongest enzyme inhibitors in our study, to the active pocket of *α*-glucosidase (Figure 5). Its aglycone formed Pi-anion interaction with the key residues including Glu276, Asp349, and Arg312; H-bond with Gln350; and Pi-alkyl with Arg439. Interestingly, rhamnosyl moiety of compound **3** also has Pi-alkyl interaction with Arg312 at its methyl group, which is the same as that of compound **2**, indicating Arg312 might be a key residue that interacted with the glycosyl groups. Among the flavonol glycosides, compounds **8** and **1** showed a relatively more powerful inhibitory effect on *α*-glucosidase, and both of their glycosyl group formed hydrogen bonds with Arg312; however, such interaction disappeared for those flavonol glycosides with poor activity, such as compounds **13** and **18** (Figure 5).

RETRACTED

### 3.6. CoMFA and CoMSIA Models Are Developed Successfully with Good Stability and Predictability

CoMFA and CoMSIA methods were applied to build 3D-QSAR models to explore how change in 3D structural features of chemical groups substituted on flavonol backbone affects *α*-glucosidase inhibitory activity. The training set with 21 structurally optimized flavonols was aligned well for the construction of the models (Figure 6(a)). Statistical parameters of both CoMFA and CoMSIA models were calculated by PLS analysis and LOO option, which are all listed in Table 2, as shown in *q*^2^ of 0.598 and 0.730, ONC of 14 and 7, SEE of 0.004 and 0.055, and *F* of 123105.135 and 1144.174, respectively, indicating the high robustness and good predictive power of the generated models. The predicted pIC_50_ values obtained via CoMFA or CoMSIA analyses, along with the actual data, of flavonols in both training and test sets, are recorded in Table 3 and depicted graphically as scatter plots (Figures 6(b) and 6(c)). In the training set, the predicted activities by either CoMFA or CoMSIA models were in line with the experimental data with *R*^2^ being 1.000 and 0.998, and in the test set, *r*^2^_pred_ is of 0.906 and 0.896 (Table 2), respectively, suggesting the constructed models were reliable with good predictability.

### 3.7. 3D Contour Maps of QSAR

CoMFA and CoMSIA models are illustrated in Figure 7 using 3D contour maps, with compound **2**, the most potent inhibitor, as the template molecule. In CoMFA, field contributions of steric and electrostatic descriptor were 55.1% and 44.9%, respectively. CoMSIA contained five descriptors including steric, electrostatic, hydrophobic, hydrogen bond donor, and hydrogen bond acceptor fields with the contributions of 11.2%, 25.5%, 13.0%, 30.2%, and 20.1%, respectively (Table 2).

RETRACTED

In CoMFA, steric field is illustrated in green and yellow contours, representing the bulky-favorable and bulky-unfavorable region, separately. A large yellow contour around C-3 position at ring C demonstrated that the presence of bulky groups in this region would decrease the activity (Figure 7(a)). It is in conformity with the results of the in vitro inhibition test on *α*-glucosidase. Compounds **21** (myricetin), **22** (quercetin), **23** (kaempferol), and **26** (isorhamnetin) had more potent inhibitory effect on *α*-glucosidase than their 3-*O*-glycosides, which include glycoside groups as bulky components substituted at position 3 of ring C (Table 1). The green counters around the rhamnosyl group of compound **2** indicated that this region containing bulky substituents would improve the activity (Figure 7(a)). It was supported by the results that compound **2**, with a galloyl moiety (bulky group) attached to the C-2^″^ position at rhamnose ring of myricitrin (compound **1**), showed significantly increased inhibitory capacity on *α*-glucosidase in comparison to that of compound **1**, whose pIC_50_ values were 5.879 and 3.110, respectively. Similarly, compound **3**, the isomer of compound **2**, with a galloyl group substituted at C-4^″^ of myricitrin, also had much stronger *α*-glucosidase inhibitory activity with a pIC_50_ value of 5.752.

As for the electrostatic contour map in CoMFA, red or blue contour separately depicted the favorable location for the electronegative or electropositive groups (Figure 7(b)). Red contours near C-3′ and C-5′ in the B ring indicated that the electronegative substituents were favored in this region. Hence, compounds **21** (3′,4′,5′-OH) and **22** (3′,4′-OH) had stronger inhibition capacities on *α*-glucosidase in comparison with compound **23** (4′-OH), as shown in the pIC_50_ values of 4.807, 4.451, and 4.149, respectively. Meanwhile, compound **21**, with two hydroxyl groups as electronegative substituents at both C3′ and C5′ of ring B, exhibited enhanced inhibitory activity than that of compound **22**, which possess just a hydroxyl group at the C3′ position. A large blue area encircling the rhamnose ring and C3 of the ring C demonstrated the introduction of electropositive groups in these areas would improve the *α*-glucosidase inhibitory effect of flavonols (Figure 7(b)). It was supported by the facts that compounds **2** and **21** showed stronger inhibition capacity against *α*-glucosidase than compound **1**. The CoMSIA model showed similar steric (Figure 7(c)) and electronic contour maps (Figure 7(d)) as the CoMFA model, confirming the importance of these two fields in the *α*-glucosidase inhibitory activity of flavonols.

RETRACTED

## 4. Discussion

Oxidative stress is closely related to the occurrence and development of a variety of chronic diseases such as DM and obesity [26]. Intake of natural antioxidants is an effective strategy to ameliorate oxidative stress in human body and contribute to prevention and treatment of chronic diseases [27]. Among the tested tissues, bayberry leaf showed the highest antioxidant activity, which can act as a potent scavenger of ROSs and has great medicinal values.

Structural elucidation of major components in Chinese bayberry leaf is essential for accurate pharmacodynamics and its further development. Six flavonols were precisely prepared and characterized from the pruned bayberry leaves, among which myricetin is the main aglycones along with different decorations including glycosylation and galloylation [18]. Compound **1** was the most abundant flavonols in leaves (9.42 mg/g FW), which is much higher than that of mature fruits (ranging from 0.01 to 0.05 mg/g FW in different cultivars) [11]. Therefore, bayberry leaves are idle materials for the mass preparation of compound **1**.

Compound **1** exhibited substantial *in vitro* antioxidant capacities by DPPH and FRAP assays and protected human keratinocytes from sodium arsenite-induced oxidative stress [28]. Compound **1** also showed great antioxidant effect in vivo, which significantly ameliorated hepatic oxidative stress in carbon tetrachloride-intoxicated mice, as shown by the decrease in lipid peroxidation and concomitant increase in glutathione level [29]. Based on such great antioxidant potential of compound **1**, its mass production from bayberry leaves by the developed protocol in the present study provides a material basis for further pharmacology development.

Additionally, to our best knowledge, compound **3** was first characterized in bayberry leaves by using LC-MS and NMR [30]. It was ever reported in *Eugenia uniflora* leaves and exhibited potent DPPH radical scavenging activity and antibacterial effect [31]. Compound **2** was the isomer of compound **3**, which was identified as compound **1** further introduced a galloyl moiety at C2^″^ or C4^″^ position, separately. As reported, compound **2** was also found in leaves of *Acacia confusa* and possessed great free radical-scavenging activity [32]. Such two compounds were also found to exert higher antioxidant effects than those of compound **1** [31, 32], indicating the enhancement on antioxidant ability of galloylation of flavonols. However, so far, there are no reports about the functions of these two compounds on oxidative stress-induced diseases such as DM and obesity. In the present study, we supplemented new evidence for the antidiabetic potential of galloylated flavonol glycosides. The developed purification protocol from bayberry leaves also provides foundation for the further study.

RETRACTED

As shown in the hundredfold decreased IC_50_ values of compounds **2** and **3** than those of compound **1**, it suggested that galloylation significantly enhanced the inhibition capacity of flavonols against *α*-glucosidase. As reported, native pectin acylated with gallic acid showed significantly enhanced antioxidant and antibacterial activities [33]. The galloylated monomeric catechins clearly showed more potent functions on improving dentin biomodification properties than nongalloylated analogues [34]. Furthermore, the galloyl moiety remarkably increased the inhibition capability of catechin against aldose reductase [35] and key digestive enzymes relevant to DM [36–38]. Here, we proved the enhancement effect of galloylation of flavonols on *α*-glucosidase inhibitory activity by comparison between compound **1** and compounds **2** and **3**. Therefore, the galloyl group might be a key pharmacophore greatly improving bioactivities of flavonoids.

Docking simulation results illustrated that the introduction of galloyl moiety altered the binding orientation of flavonols to *α*-glucosidase. Pi-conjugation was generated between the benzene ring of the galloyl group and the aromatic ring of key residues such as His279, at the active site of *α*-glucosidase. Previous reports showed that hydrogen bond interaction with His279 contributed to the stable binding of other phytochemicals and *α*-glucosidase, indicating that it was one of the key amino acid residues in the *α*-glucosidase-ligand recognition [39, 40]. In addition, intermolecular interactions involving aromatic rings play a key role in the process of chemical and biological recognition, among which pi-effects would provide a significant amount of binding enthalpy for protein-ligand binding [41]. Therefore, pi-effects generated on the galloyl group with the key residues at the active cavity of *α*-glucosidase greatly increased the flavonol-enzyme binding interactions, which might be the reason why compounds **2** and **3** exhibited much stronger *α*-glucosidase inhibitory activity.

In order to systematically explore the SAR between flavonols and *α*-glucosidase, more natural flavonols were introduced and determined enzyme inhibitory activity. Isolation of pure compounds together with determination on enzyme inhibition activity is the common way to seek for effective *α*-glucosidase inhibitor [42]. However, such workload was too large based on the huge diversity of flavonols. Construction of 3D-QSAR models is an effective way to quickly screen bioactive substances as a replacement method of experimental determination and provide guidance for new drug design [43]. Here, two 3D-QSAR models by CoMFA and CoMSIA methods were constructed with regard to the *α*-glucosidase inhibitory effect of diverse flavonols, based on the accurate data obtained from 26 flavonols. Though *α*-glucosidase inhibitory effects of certain flavonols have been reported before, IC_50_ values would make a big difference resulting from the inconformity of enzyme sources, manufacturer of standards, and measurement conditions [44]. Hence, determination in a uniform standard was beneficial for the high accuracy and predictability of the established 3D-QSAR models. Ultimately, the CoMFA and CoMSIA models concerning the *α*-glucosidase inhibitory effect of flavonols were successfully developed, which were validated to possess excellent stability and predictive ability by both internal and external methods [25]. Moreover, the introduction of two strong *α*-glucosidase inhibitors with new structural features (compounds **2** and **3**) would enhance the robustness of the models.

RETRACTED

By comprehensive analysis of 3D counter maps of both CoMFA and CoMSIA models, the metapositions of ring B favored minor and bulky groups simultaneously as well as electronegative groups. This was in agreement with our experimental data that myricetin (compound **21**) showed stronger activity than quercetin (compound **22**), followed by kaempferol (compound **23**). It demonstrated that the increasing B-ring hydroxylations enhanced *α*-glucosidase inhibition capabilities of flavonoids [20, 36]. Besides, position 3 of ring C favored minor and electropositive groups, which could explain why flavonol glycosides showed decreased *α*-glucosidase inhibitory effect than the corresponding flavonol aglycones. This unveiled that 3-*O*-glycosylation seems to decrease the antidiabetic potential of flavonoids [45]. Similar explanations are for the enhancement effect of galloyl moiety attached to the rhamnose ring by comparing compound **2** or **3** with compound **1**. Such SAR results are illustrated and summarized in Figure 8, where the galloyl group in compounds **2** and **3** is crucial for *α*-glucosidase inhibitory activity. The established 3D-QSAR models could provide valuable information for the prediction of flavonols with great antidiabetic potential.

RETRACTED

## 5. Conclusion

In conclusion, the present study precisely prepared and characterized six flavonols from bayberry leaves. Compound **2** and compound **3** exhibited much higher *α*-glucosidase inhibition activity than that of positive control acarbose. Galloylation decoration of these two compounds markedly enhanced the enzyme inhibitory activity of flavonols. Molecular docking analysis illustrated that the presence of the galloyl group altered the binding orientation of *α*-glucosidase with flavonols. Furthermore, two 3D-QSAR models constructed by CoMFA and CoMSIA were validated for a good stability and predictability on inhibition capacity of flavonols against *α*-glucosidase. Such results provide valuable information for search and design of novel *α*-glucosidase inhibitors.

## Figures and Tables

**Figure 1:** Antioxidant activity (a) and *α*-glucosidase inhibitory effects (b) of flavonol-rich methanol extracts from leaf, stem, and young fruit of Chinese bayberry and workflow of the present study (c). “M” for myricetin, “Q” for quercetin, “K” for kaempferol, “I” for isorhamnetin, “Rha” for rhamnoside, “Gal” for galactoside, and “Glu” for glucoside.

**Figure 2:** MS2 spectra of flavonols in bayberry leaf extracts. ^∗^Compounds characterized by literature information and matching with the retention time, spectrum information, and MS^n^ spectral data of commercial standards. ^#^Compounds characterized based on the fragment ion information of LC-MS, theoretical MS/MS tags, literature information, and NMR.

**Figure 3:** Dose-dependent changes in *α*-glucosidase inhibitory effects of different fractions and six purified compounds from bayberry leaves. The IC_50_ value of acarbose is 238.33 *μ*g/mL that is equal to 369.15 *μ*M.

**Figure 4:** Proposed binding poses of representative flavonols to the active pocket of *α*-glucosidase.

**Figure 5:** Schematic 2D diagram of the representative flavonols interacted with key residues within the active cavity of *α*-glucosidase

**Figure 6:** Molecular alignment (a) and plots of experimental values and predicted values of flavonols in the training set and test set by CoMFA (b) and CoMSIA (c).

**Figure 7:** Steric (a) and electrostatic (b) contour map of the CoMFA model. Steric (c) and electrostatic (d) contour maps of the CoMSIA model. Green and yellow contours represent the bulky-favorable and bulky-unfavorable region, respectively. Red or blue contour separately depicted the favorable location for the electronegative or electropositive groups.

**Figure 8:** Summary of the structure-activity relationship (SAR) of galloylated flavonols analyzed in the present study as *α*-glucosidase inhibitors. The up and down arrows represent increasing and decreasing inhibition activity, respectively.

RETRACTED

**Table 1:** Chemical structures of 26 natural flavonols tested in this study.


No.	Flavonols	Synonyms	M.W.	R_3__′_	R_4__′_	R_5__′_	R_3_	R_5_	R_7_	R_8_	IC_50_ (*μ*M)
1	Myricetin-3-*O*-rhamnoside	Myricitrin	464.38	OH	OH	OH	Rhamnoside	OH	H	H	776.93 ± 10.11
2	Myricetin-3-*O*-(2^″^-*O*-galloyl)-*α*-l-rhamnoside	—	616.10	OH	OH	OH	(2^″^-O-Galloyl)-*α*-l-rhamnoside	OH	H	H	1.32 ± 0.17
3	Myricetin-3-*O*-(4^″^-*O*-galloyl)-*α*-l-rhamnoside	—	616.10	OH	OH	OH	(4^″^-O-Galloyl)-*α*-l-rhamnoside	OH	H	H	1.77 ± 0.19
4	Quercetin-3-*O*-galactoside	Hyperoside	464.40	OH	OH	H	Galactoside	OH	H	H	1148.19 ± 47.69
5	Quercetin-3-*O*-glucoside	Isoquercitrin	464.40	OH	OH	H	Glucoside	OH	H	H	1195.95 ± 34.26
6	Quercetin-3-*O*-rhamnoside	Quercitrin	448.40	OH	OH	H	Rhamnoside	OH	H	H	1038.97 ± 5.59
7	Myricetin-3-*O*-galactoside	—	480.40	OH	OH	OH	Galactoside	OH	H	H	1161.09 ± 25.12
8	Quercetin-3-*α*-l-arabinofuranoside	Avicularin	434.30	OH	OH	H	Arabinoside (furan type)	OH	H	H	419.60 ± 2.41
9	Quercetin-3-*α*-l-arabinopyranoside^∗^	Guaijaverin	434.30	OH	OH	H	Arabinoside (pyran type)	OH	H	H	598.96 ± 16.41
10	Quercetin-3-*O*-glucuronide	Miquelianin	478.40	OH	OH	H	Glucuronide	OH	H	H	>2000
11	Quercetin-3-*O*-robinobioside^∗^	—	610.50	OH	OH	H	Robinobioside	OH	H	H	>2000
12	Quercetin-3-*O*-rutinoside	Rutin	610.50	OH	OH	H	Rutinoside	OH	H	H	>2000
13	Quercetin-3-*O*-gentiobioside	—	626.50	OH	OH	H	Gentiobioside	OH	H	H	>2000

No.	Flavonols	Synonyms	M.W.	R_3__′_	R_4__′_	R_5__′_	R_3_	R_5_	R_7_	R_8_	IC_50_ (*μ*M)
14	Kaempferol-3-*O*-rhamnoside	Afzelin	432.40	H	OH	H	Rhamnoside	OH	H	H	549.22 ± 14.40
15	Kaempferol-3-*O*-galactoside^∗^	Trifolin	448.40	H	OH	H	Galactoside	OH	H	H	837.83 ± 20.19
16	Kaempferol-3-*O*-glucoside	Astragalin	448.40	H	OH	H	Glucoside	OH	H	H	1074.57 ± 28.21
17	Kaempferol-3-*O*-rutinoside^∗^	Nicotiflorin	594.50	H	OH	H	Rutinoside	OH	H	H	>2000
18	Kaempferol-3,7-dirhamnoside	Kaempferitrin	578.50	H	OH	H	Rhamnoside	OH	Rhamnoside	H	>2000
19	Isorhamnetin-3-*O*-glucoside	—	478.40	OCH_3_	OH	H	Glucoside	OH	H	H	>2000
20	Isorhamnetin-3-*O*-rutinoside	Narcissoside	624.50	OCH_3_	OH	H	Rutinoside	OH	H	H	>2000
21	Myricetin	—	318.24	OH	OH	OH	H	OH	H	H	15.61 ± 0.34
22	Quercetin	—	302.24	OH	OH	H	H	OH	H	H	35.39 ± 2.41
23	Kaempferol	—	286.24	H	OH	H	H	OH	H	H	71.00 ± 0.20
24	Fisetin	—	286.24	OH	OH	H	H	H	H	H	86.34 ± 1.33
25	Herbacetin	—	302.24	H	OH	H	H	OH	H	OH	123.12 ± 1.57
26	Isorhamnetin^∗^	—	316.26	OCH_3_	OH	H	H	OH	H	H	319.54 ± 1.05
	Acarbose (positive control)										369.15 ± 6.18

^∗^Test set.

RETRACTED

**Table 2:** Statistical data and field contribution of 3D-QSAR models.

	CoMFA	CoMSIA
Statistics parameters		
*q*^2^	0.598	0.730
*R*^2^	1.000	0.998
ONC	14	7
SEE	0.004	0.055
*F*	123105.135	1144.174
Field contribution (%)		
Steric	55.1	11.2
Electrostatic	44.9	25.5
Hydrophobic	—	13.0
Hydrogen bond donor	—	30.2
Hydrogen bond acceptor	—	20.1
*r*^2^_pred_	0.906	0.896

CoMFA: comparative molecular field analysis; CoMSIA: comparative similarity index analysis; *q*^2^: cross-validated correlation coefficient; *R*^2^, non-cross-validated coefficient; ONC: optimal number of components; SEE: standard error of estimation; *F*: *F* test value; *r*^2^_pred_: predictive correlation coefficient.

**Table 3:** Predicted activities of flavonols in the training set and test set by CoMFA and CoMSIA.

No.	Flavonols	IC_50_ (*μ*M)	pIC_50_	CoMFA		CoMSIA	
				Pred-pIC_50_	Pred-IC_50_ (*μ*M)	Pred-pIC_50_	Pred-IC_50_ (*μ*M)
1	Myricetin-3-*O*-rhamnoside	776.93	3.110	3.111	774.46	3.163	687.07
2	Myricetin-3-*O*-(2^″^-*O*-galloyl)-*α*-l-rhamnoside	1.32	5.879	5.878	1.32	5.873	1.34
3	Myricetin-3-*O*-(4^″^-*O*-galloyl)-*α*-l-rhamnoside	1.77	5.752	5.753	1.77	5.764	1.72
4	Quercetin-3-*O*-galactoside	1148.19	2.940	2.943	1140.25	2.851	1409.29
5	Quercetin-3-*O*-glucoside	1195.95	2.922	2.923	1193.99	2.867	1358.31
6	Quercetin-3-*O*-rhamnoside	1038.97	2.983	2.984	1037.53	3.078	835.60
7	Myricetin-3-*O*-galactoside	1161.09	2.935	2.933	1166.81	2.957	1104.08
8	Quercetin-3-*α*-l-arabinofuranoside	419.60	3.377	3.376	420.73	3.401	397.19
10	Quercetin-3-*O*-glucuronide	>2000	2.666	2.667	2152.78	2.655	2213.09
12	Quercetin-3-*O*-rutinoside	>2000	2.280	2.281	5236.00	2.284	5199.96
13	Quercetin-3-*O*-gentiobioside	>2000	2.207	2.206	6223.00	2.183	6561.45
14	Kaempferol-3-*O*-rhamnoside	549.22	3.260	3.26	549.54	3.235	582.10
16	Kaempferol-3-*O*-glucoside	1074.57	2.969	2.969	1073.99	2.932	1169.50
18	Kaempferol-3,7-dirhamnoside	>2000	2.097	2.097	7998.34	2.112	7726.81
19	Isorhamnetin-3-*O*-glucoside	>2000	2.489	2.485	3273.41	2.522	3006.08
20	Isorhamnetin-3-*O*-rutinoside	>2000	2.097	2.097	7998.34	2.115	7673.61
21	Myricetin	15.61	4.807	4.806	15.63	4.833	14.69
22	Quercetin	35.39	4.451	4.452	35.32	4.385	41.21
23	Kaempferol	71.00	4.149	4.144	71.78	4.092	80.91
24	Fisetin	86.34	4.064	4.065	86.10	4.119	76.03
25	Herbacetin	123.12	3.910	3.914	121.90	3.922	119.67
9	Quercetin-3-*α*-l-arabinopyranoside^∗^	598.96	3.223	3.422	378.44	3.580	263.03
11	Quercetin-3-*O*-robinobioside^∗^	>2000	2.428	2.281	5236.00	2.284	5199.96
15	Kaempferol-3-*O*-galactoside^∗^	837.83	3.077	3.138	727.78	2.951	1119.44
17	Kaempferol-3-*O*-rutinoside^∗^	>2000	2.114	2.367	4295.36	2.308	4920.40
26	Isorhamnetin^∗^	319.54	3.495	4.092	80.91	3.959	109.90

^∗^Test set.

RETRACTED

## Data Availability

The authors confirm that the data supporting the findings of this study are available within the article.

## Supplementary Materials

Supplementary Materials Supplementary Figure 1: high-resolution mass identification of purified compound **2**. Supplementary Figure 2: high-resolution mass identification of purified compound **3**. Supplementary Figure 3: NMR identification of purified compound **2** in DMSO-*d6*. Supplementary Figure 4: NMR identification of purified compound **3** in DMSO-*d6*.
